# An Efficient Identification of Security Threats in Requirement Engineering Methodology

**DOI:** 10.1155/2022/1872079

**Published:** 2022-08-18

**Authors:** R. Subha, Anandakumar Haldorai

**Affiliations:** Department of Computer Science and Engineering, Sri Eshwar College of Engineering, Coimbatore, Tamil Nadu, India

## Abstract

Today, we completely rely on Information Technology (IT) applications for every aspect of daily life, including business and online transactions. In addition to using these IT-enabled applications for business purposes, we also use WhatsApp, Facebook, and a variety of other IT applications to communicate with others. However, there will undoubtedly be a drawback to every benefit. Since everything is linked to the Internet, there are many opportunities for security to be compromised. To address this, we are working to identify security threats early on in the software development process, specifically during the requirements phase. During the requirement engineering process, an engineer can recognize the security specifications in a more structured manner to create threat-free software. In our research work, we suggest the Identification of Security Threats during Requirement Engineering (ISTDRE) technique for detecting security risks throughout the requirement engineering process. The four points that make up this ISTDRE technique are Hack Point (HP), Speculation Point (SP), Trust Point (TP), and Reliable Point (RP). The new ISTDRE methodology will be validated using a case study of an ERP system involving two currently used methodologies: Model Oriented Security Requirements Engineering (MOSRE) and System Quality Requirements Engineering (SQUARE).

## 1. Introduction

Since we are moving into a digital world, data handling systems, which process information, are in high demand. The systems are vital since they are capable of processing data effectively in a timely manner. Due to this, everyone is in need of software security that will protect their data from hackers or threats [1]. So, to procure software that has quality security systems, we should have the appropriate security requirements engineering. To overcome this issue, we need to be more concerned about the security issue during the first stage of software development, which is the requirement phase. During this phase, we need to shape the security systems by including security procedures and actualizing them effectively by using the security requirement engineering process [2].

There are so many security breaches nowadays in all the software. Recently, a popular videoconferencing app also had a security breach, and many people were affected by it. So, in order to avoid this kind of threat to an organization, everyone is more concerned about the security system that protects its software from hackers. Everyone is surfing over the Internet and running 24/7 to find a security system that has a sufficient amount of security that no hacker can break it. It is vital to acquire software that would not be exploited by hackers and any harmful processes. That level of the softwares are being created by several software experts, lecturers, or authors who have spent their time, heart, and soul in building it. We must now figure out how to obtain the security requirement engineering. We all know that the 1^st^ phase of software development is requirements engineering. In the requirement engineering process, we will define the needs or conditions to meet the Partner goal. In that, there are 2 types of requirements engineering, which are functional and nonfunctional. Our security requirement engineering comes under nonfunctional requirement engineering, which is a precious step to getting quality software [3]. We should put more emphasis on security requirements engineering in order to produce high-quality software. To attain the goal of the user without a security breach, we need to get the security requirement [4] from the Partner which is not an easy task to do. To get that from the Partner, we should explain what requirement engineering is all about. When it comes to the digital world, the security requirements will be broad to protect sensible information and important data.

In order to get to the initial phase of the software development cycle, that is, during the requirement engineering process, we have suggested the security requirement engineering techniques in this paper. Usually, during the requirement engineering process, the requirement engineer will concentrate more on functional requirements, which are more essential for the software development process, but they fail to cover the security requirements engineering while the requirement engineer gets only the functional requirements engineering from the user. The majority of requirement engineers are proficient in functional requirement engineering. When it comes to security requirements engineering, most of the engineers have less knowledge about it and even the partners of the software do not know much about it. But the stimulation of the security engineering requirements from the user is quite a hectic task for the requirement engineer. Sometimes the partners will recommend the most valuable resource in the software that needs to be safeguarded [5]. During this time, the requirement engineer will investigate the threads and classify them separately, after which the requirement engineer will investigate and develop the security requirements engineering to protect the software from hackers.

As previously stated, most requirement engineers are unaware of security requirement engineering and its entire process, resulting in ambiguous information. As a result, our goal is to obtain well-assembled security requirements engineering approaches to protect our software from hackers. This assembled security requirement engineering will be a big help for the requirement engineer to produce software that will not be hacked by hackers. And we are going to use the list of steps in the “Identification of Security Thread during Requirement Engineering (ISTDRE)” approach to identify the security thread in the first phase of the software development cycle, that is, during the requirement engineering process. The remaining sections are organized as follows: Section 2 contains Literature Review, Section 3 introduces an Identification of Security Threats during Requirement Engineering (ISTDRE) Technique, Section 4 discusses the Thematic Study of ERP system, Section 5 contains Result and Discussion, and this paper concludes with future research in Section 6.

## 2. Literature Review

Our paper is not the first of its kind to demonstrate the importance of software security in the requirement engineering process. There have been many researchers who have done extensive research to improve software security through various techniques. In this section, we are going to discuss the various techniques that have already been proposed by different researchers. The first technique we are going to discuss is SIREN [6], which reuses the requirements, and the other proposed technique is the extension of Unified Modeling Language [SIREN], which has a multilevel security system and has access dominance. In another technique, the model-driven security method, they merged the Unified Modeling Language with its Secure Unified Modeling Language to create software that cannot be hacked by hackers.

One of the prominent researchers [7] described the new technology known as system-theoretic analysis, which explains how we can get the security requirements engineering by visiting the client organization and getting information from the business person. Another brilliant researcher [8] described another technique, the Troops approach, which is based on identifying each and every piece of information about the software that is from the requirement engineering process and then moving into the organization and analyzing the software where it is being used and constructing the software so that it cannot be hacked by the hackers.

Another analyst [9] proposed a strategy dependent on issue outlines and misuse outlines for security prerequisite elicitation. They utilized issue edges to construct a security list and to speak to security prerequisites, while the maltreatment outlines are utilized for danger demonstrating. The next researcher [10] proposed the STS approach for modeling and reasoning about security requirements. In this approach, security requirements are identified by the STS-ml requirements modeling language. The requirements models of STS-ml have a formal semantics which allows automated reasoning for detecting possible conflicts among security requirements as well as conflicts between security requirements and actors' business policies.

Let us discuss another research paper [11], which created a Discovering Goals for Security (DIGS) structure that models the key substances in data security, counting resources, and security objectives. Another researcher [12] proposed a gauges-based procedure, named SREP (Security Requirements Building Process), that manages the security prerequisites during the beginning periods of programming improvement in an orderly and natural way.

Now let us look into another strategy proposed by a veteran author. [13] suggested that before developing the software, we need to check the history of the software and use the security requirements engineering to develop software that cannot be hacked by hackers. Recently, many researchers have developed so many strategies to develop software by developing security during the requirement engineering process itself. The latest invention is the Requirements Engineering Readiness Model, which lets firms check the security requirement engineering process.

Not every paper that is published to enhance the security of software describes the software development process. Sometimes the paper may deviate from its main objective (i.e., security requirement engineering) and focus more on the requirement engineering process, which looks into functional requirement engineering. More recent papers that use the methodology, such as MSRA, Tropos, SQUARE, and SRERM, concentrate on security requirements engineering to protect software from hackers [14].

## 3. Introduction of Identification of Security Threats during Requirement Engineering (ISTDRE) Technique

Now let's investigate our strategy Identification of Security Threats during Requirement Engineering (ISTDRE) in brief.

### 3.1. Identification of Security Threats during Requirement Engineering (ISTDRE) Technique

In our Identification of Security Threats During Requirement Engineering (ISTDRE) Technique, we go through the series of processes in which we will be getting the security requirements engineering of the software from the Partner (P) of the firm in order to get a precise and reliable requirement because they know what the software requires and they may also be aware of the loopholes where hackers will try to hack the software. Our ISTDRE strategy collects a set of security requirements from our partners, and then, they define their own requirements to protect the software from viruses and hackers. During this process, the requirement engineer will check the risks associated with the development of the software and then they will develop the plan to overcome those issues.

The above Figure 1 represents the security requirements engineering concept model [14] for the proposed Identification of Security Threats during Requirement Engineering (ISTDRE) technology. It is to be noted that the software which is being developed may have more than one partner, and it is not necessary that all the partners be involved in the security of the software. These partners also have knowledge of the valuable resource (VR) that is to be protected from the hackers. We will diagnose the Partners (P) and arrange them based on their abilities in our ISTDRE. Since in our ISTDRE strategy the input of the Partners (P) is very important, we should consider their input valid and proceed with the software development.

The valuable resource (VR) is the important tool that is to be secured from hackers. To show the VR of the software product, the partners will help the requirement engineer. Since we all know that our ISTDRE strategy has a series of operations, every operation is similarly essential. The above Figure 2 stands for the activity diagram of the Identification of Security Threats during Requirement Engineering (ISTDRE) technology [14].

So, our requirement engineer cannot just simply avoid any of the operations and continue with the next operation because there will be connectivity between the operations if they skip any of those mentioned in the security requirement engineering, which was designed by the requirement engineer with the help of the partners who were well aware of the security of the software product [15].

### 3.2. Measures of Identification of Security Threats during Requirement Engineering (ISTDRE)

As we have already discussed, lots of steps are involved in our Identification of Security Threats during Requirement Engineering (ISTDRE) strategy. In this chapter, we are going to discuss each and every step, and then, we are going to discuss the inputs we got from the partners and what all the steps we constituted by taking in the suggestions or requirements given by the partners during our security requirement engineering process (Table1. Let's illustrate one by one for easy understanding [14].

**Step 1 .**

Recognizing system targets.

**Step 2 .**

Recognizing and identifying the Partners.

**Step 3 .**

Approved the targets.

**Step 4 .**

Recognizing VR.

**Step 5 .**

Examination of security threats (Hack Point [HP], Trust Point [TP], Speculation Point [SP], and Reliable Point [RP]).

**Step 6 .**

Recognizing and classifying the threat.

**Step 7 .**

Hazard valuation and recognizing.

**Step 8 .**

Security requirement evocation.

**Step 9 .**

Security requirement certification.

**Step 10 .**

Security requirement stipulation record.

#### 3.2.1. Recognizing System Targets

The objective of the Identification of Security Threats during Requirement Engineering (ISTDRE) strategy's 1^st^ step is to recognize system targets [14]. The targets will be set by the partner with whom we are developing the software. The targets, which are most important for the software system, are collected from the partners by the requirement engineer [16] during the requirement engineering process, which is the 1^st^ phase of the software development life cycle, and then, while getting the requirement from the partner, the requirement engineer will record the targets indicated by the partner either orally or in a written document. And to achieve the targets set by the Partner, the requirement engineer will write so many approaches by which the requirement engineer can satisfy all the needs of the Partners, which is his utmost aim [17]. We can use any of the strategies (interrogation, creative thinking, examining, and meeting interrogation) to get the suggestion from the Partner. And then, the result of the 1^st^ step, which is recognizing system targets, will be “Catalogues of System Objectives.”

#### 3.2.2. Recognizing and Identifying the Partners

Recognizing and identifying the partners is the second and most important part of our Identification of Security Threats during Requirement Engineering (ISTDRE) strategy. In this step, the requirement engineer should identify the partners based on their importance in the software development life cycle [18]. The software authorities may be one or more during the partner identification. In the case of one, he will be the most important person and we have to get the requirements from him, even the security requirements engineering, because he might be the only person associated with the firm and he might be aware of the end product [19]. For example, if we have 2 or many partners in the organization, we must recognize the partners based upon their importance level for the software development process. For example, the partner may be classified into 3 types: most important, important, and less important. The most important partners are those we should not miss out on during the entire software development process. Next are the important partners; if we miss them, then the software development process will become boring, and the least important partners, if we miss their suggestion, will not create any major drawback in the system [20].

#### 3.2.3. Approved the Targets

Following the recognition of the partners, our next goal is to confirm the targets they provided us during the requirement engineering process. In this step, we need to converse with all the partners and the concerned person responsible to get a clear indication [21]. We should be 100% sure that we had documented the targets which were given by partners are correct, and we should get a statement from all the partners that the above said targets were their only goal and there was no change in them. We should make a record of it just to be clear on what they want or what the target is. We can use any of the strategies (interrogation, creative thinking, examining, and meeting interrogation) to get the suggestion from the partner [22].

#### 3.2.4. Recognizing Valuable Resources (VR)

Our main objective of the paper is to secure valuable resources from hackers. In order to attain this, we are doing security requirement engineering during the 1^st^ phase of the software development life cycle, that is, during the requirement engineering process. So, this is the most important step. We must be very keen on this step. We have to check with all the partners or the most important partner who is more concerned about the security of the software. The valuable resources can be money, passwords, user data, personal information, etc. It can be of any type. We have to get this from the partner, and we have to regularize the security check for these valuable resources (VR). After conversing with the partners of the organization, we have to give preference based on the importance of the VR and then give them security based on it.

#### 3.2.5. Examination of Security Threats

This requires the use of several strategies, and it is the most important step in the security requirement engineering process. In this step, we are going to devise a plan on which technique will handle which type of threat and how to protect our VR and the whole software from those threats. For this, we have devised 4 approaches: Hack Point (HP), Trust Point (TP), Speculation Point (SP), and Reliable Point (RP) [23].

*(1) Hack Point (HP)*. Whenever there is a software or application which gets input from the user's end, then there will be HP definitely. We need to concentrate more on these Hack Points. The Hack Points may be the login page or any page that gets input from the end user. These points are the deficiencies of the software because most of the Hackers try to hack the software from those points [24].

*(2) Trust Point (TP)*. Trust Point is nothing but the trustable source of the software. For example, whenever we develop a web page or software, we give full authorization to the admin. So, the admin is the trustable source. Hackers use this point, and he pretends to be an admin, and then, he tries to enter into the software and hacks the software. As a result, the requirement engineer must be aware of such issues and strengthen the security checks in that TP [25].

*(3) Speculation Point (SP)*. After the software's development, there will be some other chance for the hacker to crack the software. So, this Speculation Point gives us where there will be issues that it has to care about. For that, the programmer has to recheck the software after the development and before the implementation process, and if there are any issues, he must resolve them before he can implement the software in the client's place.

*(4) Reliable Point (RP)*. The Reliable Points (RP) are those points upon which the software wholly relies upon after the implementation of the software. For example, in all organizations, every piece of software or web page depends upon the server. So, we must secure our software at the Reliable Point (RP) which might be the point for the hacker to get into the software.

#### 3.2.6. Recognizing and Classifying the Threat

When we have finished examining threats such as where they might occur or from which point they will occur, the next step is to recognize and classify the thread that attempts to harm the software. During this process, we will end up finding a number of threats. The most important step is determining which threat will affect our software. To find this, there are a number of strategies, among which threat patterning is the most important of all. In this threat patterning, we will look into the background of the threats that hit the software, and then, we have to check the types of threats that attacked the software earlier. To get this in our strategy also, we are going to use Microsoft's STRIDE (Spoofing, Tampering, Repudiation, Information Disclosure, Denial of Service, and Elevation of Privilege) method.

#### 3.2.7. Hazard Valuation and Recognizing

After recognizing the threat, we are now moving into Hazard Valuation and Recognizing through which we are going to rate the identified threat found in the previous step. You know that we may end up recognizing so many threats in the previous step, and you all know that the elimination of all the found threats is not a feasible option because we may need to spend so much money on it. So, in order to overcome this issue, in this step, we are going to rank the threats based on their harm level. That is, we must first eliminate the threat that will cause more harm to the software and we can avoid the threat that will cause less harm or negligible harm to the software.

Hazard to the software = Possibility ^*∗*^ Harmful level of the threat. (If there is a more harmful threat, then there is more hazard to the software). Even so, we can assess the risk by using Microsoft's DREAD Risk assessment model [26]. DREAD_Risk_Value = (Hazard + Replicate + loss in quality + Impacted End Users + Detectable)/5.

#### 3.2.8. Security Requirement Evocation

Once we are done with the Hazard Valuation and Recognizing, we will move into the next step, which is Security Requirement Evocation. As we had learned in the earlier step, we will rank the threats and first we will eliminate the threat which is the most harmful to the software, and then, we will move on to the next important threat to be eliminated. In this step, our objective is to make the security requirement engineer aware of the threat dictionary that will help them identify the threat easily.

#### 3.2.9. Security Requirement Certification

In the earlier step, we had done the Security Requirement Evocation, in which we used the threat dictionary and identified the threats. We finally ranked the threats based on their importance level, and then, we eliminated the threat that is most important to harm the software. As we discussed earlier, the elimination of all threats is not important. We can eliminate the threat that is more harmful and avoid the elimination of the threat that is not harmful.

#### 3.2.10. Security Requirement Stipulation Record

This is the final step in our Identification of Security Threats during Requirement Engineering (ISTDRE) strategy. In this step, we must document the opinions of all the partners by using various types of documentation, such as affirmations, questions, denials, and problems. [27] The requirements engineer will verify that the requirements given by the partners are valid and then he will record them in a written document which will be sent to the programmer for developing the software. So, this is the most important step. We must verify that the requirements mentioned in the document are correct before sending it to the developer.

## 4. Thematic Study

### 4.1. Enterprise Resource Planning (ERP) System

This ERP implementation technique will be used to implement our Identification of Security Threats during Requirement Engineering (ISTDRE) strategy because most of the researchers like Nah and Lou have mentioned that this technique is the most prosperous and has the highest success rate [28, 29]. In our thematic study, we are going to implement the Hospital ERP systems, which have all the information like Doctor, Patients, Staff, lab, and Specialist Department. You all know that we are going to utilize the ERP system and most of the vendors use the Java/XML strategy [30].

### 4.2. Execution of the Case Study

In this step, we are going to implement all the steps of the ISTDRE strategy for the hospital ERP system. We are not going to skip any of the ISTDRE strategy, and we are going to implement it step-by-step to prove how effective our ISTDRE strategy is.

#### 4.2.1. Recognizing System Targets

The Identification of Security Threats during Requirement Engineering (ISTDRE) strategy's first step is Recognizing System Targets. The targets will be set by the Partner for whom we are developing the software. The targets, which are most important for the software system, are collected from the Partners by the requirement engineer during the requirement engineering process, which is the 1^st^ phase of the software development life cycle, and then, while getting the requirement from the Partner, the requirement engineer will record the targets indicated by the Partner either orally or in a written document. We can use any of the strategies (Interrogation, Creative Thinking, Examine, and Meeting) to get the suggestion from the Partner. Let us look into the Targets of the hospital ERP system in the below table (Table 2) [14].

#### 4.2.2. Recognizing and Identifying the Partners

Recognizing and identifying the Partners is the second and most important part of our Identification of Security Threats during Requirement Engineering (ISTDRE) strategy. In this step, the requirement engineer should identify the partners based on their importance in the hospital ERP system. We must recognize the Partners based upon their importance level for the software development process. For example, the partner may be classified into 3 types: most important, important, and less important. The most important partners are those whom we should not miss out on during the entire software development process. Next are the important Partners; if we miss them, then the software development process will become boring, and lastly, the least important partners; if we miss their suggestions, they will not create any major drawback in the system. Let us look at the preference of each person [14] in the hospital ERP system in Table 3.

#### 4.2.3. Approved the Targets

After recognizing the partners, our next goal is to confirm the targets they provided us during the hospital ERP system requirement engineering process. In this step, the concerned ERP software professional is responsible for clearly indicating that the target is correct and there is no ambiguity.

#### 4.2.4. Recognizing Valuable Resources (VR)

The primary goal of this paper is to protect valuable resources (VR) from hackers. In order to attain this, we are getting the security requirements engineering of the Hospital ERP system. So, this is the most important step. We must be very keen on this step. After conversing with the Partners of the organization, we have to give preference based on the importance of the VR and then give them security based on it [14]. Look at Table 4 where we listed it.

#### 4.2.5. Examination of Security Threats

In this step, we are going to devise a plan on which technique will handle which type of threat and how to protect our VR and the whole software from those threats. For this, we have devised 4 approaches: Hack Point (HP), Trust Point (TP), Speculation Point (SP), and Reliable Point (RP).

*(1) Hack Point (HP)*. If we are getting the input from the user end for the hospital ERP system, then there will be HP definitely. We need to concentrate more on these Hack Points. (Table 5) indicates the HP of the hospital ERP system [14].

*(2) Trust Point (TP)*. Trust Point is nothing but a trustable source. For example, whenever we develop a web page or software, we give full authorization to the admin [14]. So, in the hospital ERP system, the Chairman is the trustable source. (Table 6) depicts the TP of the hospital ERP system.

*(3) Speculation Point (SP)*. The Speculation Point gives us an idea of what issues there will be for which it has to care about. For that, the programmer has to recheck the software after the development and before the implementation process, and if there are any issues, he must resolve them or else he will face some issues during the implementation of software in the client's place (Table 7), which depicts the SP of the hospital ERP system [31].

*(4) Reliable Point (RP)*. The point which the software wholly relies upon after the implementation of the software is known as the Reliable Point (RP).  Table 8 depicts the RP of the hospital ERP system.

#### 4.2.6. Recognizing and Classifying the Threat

.  Table 9 depicts the threats of the Hospital ERP system.

#### 4.2.7. Hazard Valuation and Recognizing

You are aware that we may end up recognizing a large number of threats in the previous step, and you are all aware that eliminating all discovered threats is not a feasible recommendation because it may necessitate a significant financial investment. (Table 10) depicts the threat with the hazard value [14]. So, in order to overcome this issue, in this step, we are going to rank the threats based on their harm level, which means that we must first eliminate the threat that will cause more harm to the software, and we can avoid the threat that will cause less harm or negligible harm to the software.

#### 4.2.8. Security Requirement Evocation

Once we are done with the Hazard Valuation and Recognizing, we will move into the next step, which is Security Requirement Evocation [14]. As we had learnt in the earlier step, we will rank the threats, and first, we will eliminate the threat which is the most harmful to the software, and then, we will move on to the next important threat to be eliminated.  Table 11 depicts the security requirements of the hospital ERP system.

#### 4.2.9. Security Requirement Certification

As we discussed earlier, the elimination of all threats is not important. We can eliminate the threat that is more harmful and avoid the elimination of the threat that is not harmful.

#### 4.2.10. Security Requirement Stipulation Record

In this step, we must document the opinion of all the partners by using various types of documentation, such as affirmations, questions, denials, and problems. The requirement engineer will verify that the requirements given by the partners are valid, and then, he will record them in a written document, which will be sent to the programmer for developing the software.

## 5. Result and Discussion

As we already mentioned in our paper, we are going to compare our ISTDRE technique with the Model Oriented Security Requirements Engineering methodology and System Quality Requirements Engineering methodology in this chapter.

### 5.1. Examining Model Oriented Security Requirements Engineering (MOSRE) and Identification of Security Threats during Requirement Engineering Technique

In this step, we are going to examine Model Oriented Security Requirements Engineering and Identification of Security Threats during Requirement Engineering (ISTDRE) technique for which we are going to implement the abovementioned 2 techniques and find which is best. For that, we are going to choose the paper [32] because they have used Model Oriented Security Requirements Engineering in the E-Health system development to examine the valuable resources, threats, and other impacts. Look at Table 12, in which we compared both the tables and we proved that the result obtained from ISTDRE technology [14] is better than the result obtained from Model Oriented Security Requirements Engineering.

#### 5.1.1. Comparing the Model Oriented Security Requirements Engineering and Identification of Security Threats during Requirement Engineering Technique Using DREAD Risks Value

As we all know the fact, we need to eliminate the thread which is more harmful, so it is important that whatever the technique we use should eliminate the threat which is more harmful and protect our system from hackers. So, we are going to compare our technique (ISTDRE) with the already existing Model Oriented Security Requirements Engineering and prove that our technique will eliminate all the threat which is more harmful.

We have used the most important threat that will occur when the hackers try to hack the software. And in this graph (Figure 3), we have listed out the 10 most common threats in decreasing order, which have more DREAD Value, 10, and then, the threat which has the least value is listed last. Let's recollect the DREAD Value of all the threats that we have learnt about in Table 10. The threat is more harmful if the DREAD Value is high and less harmful if the DREAD risk value is low.

In that step, we identified the DREAD Value of each threat. That is, threat “User give hostile Structure Query Language (SQL) information” has the DREAD risk value of “10,” threat “Entering the DB” has the DREAD risk value of “10,” threat “ERP System Crashing” has the DREAD risk value of “10,” threat “Exposing the user information” has the DREAD risk value of “9.2,” threat “Falsification of User Information” has the DREAD risk value of “9.2,” threat “Hacking Sign in page of the Admin” has the DREAD risk value of “7.6,” threat “Removing the account of the user” has the DREAD risk value of “7.6,” threat “Entering without Sign in” has the DREAD risk value of “7.6,” threat “Exposure of sign in information” has the DREAD risk value of “6.6,” threat “Notification of Message is blocked” has the DREAD risk value of “6.4,” threat “Unpermitted Access” has the DREAD risk value of “5.2,” and threat “Hack of Session ID” has the DREAD risk value of “3.8.”

As shown in the graph above, our technology ISTDRE eliminated the threat that was more harmful to the software, and not only that but also our technique eliminated 8 of the 10 most common threats that occur to the software system. The MOSRE technique eliminates only the 3 threats out of the 10 most common threats, which allows the rest of the 7 threats to attack the software system. Hence, we prove that our proposed ISTDRE technique is more efficient in eliminating the threats and more efficient than SQUARE.

### 5.2. Examining System Quality Requirements Engineering and Identification of Security Threats during Requirement Engineering Technique

In this step, we are going to examine System Quality Requirements Engineering and Identification of Security Threats during Requirement Engineering. For this, we are going to implement the abovementioned 2 techniques and find which is best. For that, we are going to choose the System Quality Requirements Engineering (SQUARE): Case Study on Asset Management System, Phase II paper where they showed the result of SQUARE. In that, they evoked the 9 security requirements. But after referencing the evoked requirements, they chose only 5 requirements, that is SQ1, SQ2, SQ6, SQ7, and SQ8. Take a look at the table below (Table 13), where we have given the comparison of the System Quality Requirements Engineering and Identification of Security Threats during Requirement Engineering techniques. It clearly shows that our Identification of Security Threats during Requirement Engineering technique (ISTDRE) technique is far better than the System Quality Requirements Engineering technique, and it evokes more security requirements.

#### 5.2.1. Comparing the System Quality Requirements Engineering (SQUARE) and Identification of Security Threats during Requirement Engineering Technique Using DREAD Risk Value

So, we need to eliminate the thread that is more harmful, so it is important that whatever technique we use should eliminate the threat that is more harmful and protect our system from hackers. So, we are going to compare our technique (ISTDRE) with the already existing System Quality Requirements Engineering and prove that our technique will eliminate all the threats that are more harmful.

We have used the most important threat that will occur when hackers try to hack the software. And in this graph (Figure 4), we have listed out the 10 most common threats in decreasing order, which have more DREAD Value, and then, the threat which has the least value is listed last. Let's recollect the DREAD Value of all the threats that we have learnt about in Table 10. The threat is more harmful if the DREAD value is high and less harmful if the DREAD risk value is low.

In that step, we identified the DREAD Value of each threat. That is, threat “User give hostile Structure Query Language (SQL) information” has the DREAD risk value of “10,” threat “Entering the DB” has the DREAD risk value of “10,” threat “ERP System Crashing” has the DREAD risk value of “10,” threat “Exposing the user information” has the DREAD risk value of “9.2,” threat “Falsification of User Information” has the DREAD risk value of “9.2,” threat “Hacking Sign in page of the Admin” has the DREAD risk value of “7.6,” threat “Removing the account of the user” has the DREAD risk value of “7.6,” threat “Entering without Sign in” has the DREAD risk value of “7.6,” threat “Exposure of sign in information” has the DREAD risk value of  “6.6,” threat “Notification of Message is blocked” has the DREAD risk value of “6.4,” threat “Unpermitted Access” has the DREAD risk value of “5.2,” and threat “Hack of Session ID” has the DREAD risk value of “3.8.”

As shown in the graph above, our technology ISTDRE eliminated the threat that was more harmful to the software and not only that but also our technique eliminated 8 of the 10 most common threats that occur to the software system. The SQUARE technique eliminates only 4 threats out of the 10 most common threats, which allows the rest of the 6 threats to attack the software system. Hence, we prove that our proposed ISTDRE technique is more efficient in eliminating the threats and more efficient than SQUARE.

## 6. Conclusion

We reviewed the Identification of Security Threats during Requirement Engineering (ISTDRE) method, and we agreed to analyze the product's security demands at the first phase of the software development life cycle, which is the requirement engineering stage. As stated in the abstract, we began with an introduction before moving on to the requirement process and verifying the previous techniques used to improve the security of the program. In the second chapter, we then looked at techniques that were already in use. As you may have noticed, the current technique we employ is more complex because it employs a repetitive approach to identify new security requirements. In contrast, our ISTDRE technique employs a straightforward procedure that even nontechnical people can use to increase the security of the software system. After examining the methods already in use, we turned to our ISTDRE plan in the third chapter. In our technique, we gave consideration to each danger, eliminating the one that would inflict the most harm to the program first before moving on to the one that would cause the least damage. In order to safeguard the program from hackers, we had designated the Hack Point (HP), Trust Point (TP), Speculation Point (SP), and finally the Reliable Point (RP). Then, we went on to the fourth and fifth chapters, where we put our strategy—which we had learned about in the third chapter—into practice. Here, the security requirement engineering was done sequentially, without missing a beat.

Finally, we demonstrated that our ISTDRE method was significantly superior to the System Quality Requirements Engineering (SQUARE) and Model Oriented Security Requirements Engineering (MOSRE) strategies because it elicited the most suitable and comprehensive security requirement engineering. Following this, we must put our approach into practice in a real project. As a further improvement, we must create the foundation for our approach to achieve the security requirement engineering for all projects utilizing our ISTDRE approach.

## Figures and Tables

**Figure 1:** ISTDRE security requirement engineering concept model.

**Figure 2:** ISTDRE activity diagram.

**Figure 3:** Comparing the MOSRE and ISTDRE technique using DREAD risk value. Note: in the above graph, 100 shows that the threat is eliminated completely, and 0 means the threat is not eliminated. Threats are arranged in a decreasing order of DREAD risk value.

**Figure 4:** Comparing the SQUARE and ISTDRE technique using DREAD risk value. Note: In the above graph, 100 shows that the threat is eliminated completely, and 0 means the threat is not eliminated. Threats are arranged in a decreasing order of DREAD risk value.

**Table 1:** ISTDRE technique steps.

Step	Members	Strategy	Intake	Outcome
Recognizing system targets	Requirement engineer, client	Interrogation, creative thinking	Aim	System objective
Recognizing and identifying the Partners	Requirement engineer	Examine	System objective	Partners
Approved the targets	Requirement engineer, partners	Meeting	System objective	Approved the targets
Recognizing VR	Requirement engineer, partners	Interrogation	Partners resource	Precious resource
Examination of security threats	Requirement engineer, security expert	Security attack examining	Precious resource	HP, TP, SP, and RP
Recognizing and classifying the threat	Requirement engineer	STRIDE examining	HP, TP, SP, and RP	Classified and order of preference
Hazard valuation and recognizing	Requirement engineer, hazard manager	DREAD risk assessment technology	Classified and order of preference	Threats
Security requirement evocation	Requirement engineer	Threat dictionary	Threats	Security requirements
Security requirement certification	Requirement engineer, security expert	Examine	Security requirements	Important security requirement
Security requirement stipulation record	Requirement engineer	Recording	Important security requirement	Security requirement stipulation record

**Table 2:** Recognizing system targets for hospital ERP.

Target ID	Explanation
T1	All the secret information has to be protected when the hospital ERP system is installed on the web server.
T2	The next target is to install the hospital ERP safely on the DB server (database).
T3	We should use the firewall to protect the DB server from unauthorized access through the Internet.
T4	We should use the firewall to protect the web server from unauthorized access through the Internet.
T5	For straight entry, hypertext transfer protocol secure and hypertext transfer protocol ports are only to be permitted.
T6	Transmission between the database server and the web server should take place over a secure network.
T7	We should use hypertext transfer protocol secure to deploy the hospital management system.

**Table 3:** List of possible stakeholders with their significance for college ERP system.

S. No	Name	Importance	Type
1.	Chairman	Most important	Management
2.	Dean	Most important	
3.	Chief doctor	Important	

4.	Auditor	Most important	Marketing
5.	Purchasing executive	Most important	
6.	Inpatients	Important	
7.	Outpatients	Most important	

8.	ERP project manager	Most important	Information system
9.	DB admin	Most important	
10.	Programmer	Most important	
11.	Networking team	Important	

**Table 4:** Identified assets of the college ERP system.

Value resource ID	Name	Description
VR1	Patient, doctor, and admin	The value resource that relates to a patient, doctor, and admin
VR2	Patient's login data	The patient's credentials: username and password
VR3	Doctor login data	The doctor's credentials: username and password
VR4	Admin login data	The admin's credentials: username and password
VR5	Patient's personal data	The personal data that the patient enters, such as patient record
VR6	Doctor's personal data	The personal data that the doctor, such as doctor record and assets
VR7	System	Value resource that relates to the importance of the system
VR8	Accessibility of ERP system	If the hospital ERP system goes down, patient/and doctor cannot request or receive quotes.
VR9	Procedure	Value resources that relate to the process of running the web application
VR10	Request	Value resources that relate to the web application
VR11	Login	The web session associated with a logged-in patient, doctor, or admin
VR12	Backend DB session	The ability to interact with the database that stores, patient's data, doctor's data, and login credentials
VR13	Patient fee details	The patient's fee record must be secure. Manipulation of the data causes loss in data.
VR14	Doctor salary details	The doctor's salary record must be secure. Manipulation of the data causes loss in data.
VR15	Message notification	The message notification contains the information for patients and doctors
VR16	Audit data	Attackers might try to attack the system without being logged or audited
VR17	Access to the record	Authorized people only able to view the record

**Table 5:** Identified hack points (HP).

HP ID	Hack point (HP)	Explanation
HP1	Hypertext transfer protocol secure (HTTPS)	HTTPS port that the web server listens on
HP2	Access page	Page for patients or doctor to create an access and perform an access to the site to begin requesting or reviewing records
HP3	Create access function	Creates a new patient or doctor access
HP4	Access to site function	Compares authorized person login details to those in the DB and if credentials match, create a new session
HP5	Entry page	In this page, doctors' and patients' personal data will be entered into the DB.
HP6	Recover data function	Permit the allowed person to recover the DB.
HP7	Presenting data function	Permit admin to recover the doctor and patient data
HP8	Admin evolution page	Permit admin to recover the doctor and patient demand
HP9	Recover data function	Recover doctor and patient data
HP10	Presenting data function	Presenting any data information for the student or staff
HP11	List demand function	Lists requests are ready for examination.
HP12	DB listening ports	Permit the DB to be used remotely by authorized persons
HP13	DB stored procedures	Recover and save information in the DB
HP14	Access process	Build access page for permitted persons
HP15	Removing access process	Sign out from the hospital ERP system
HP16	Store user data procedure	Used to store user data from the entry page of the ERP system
HP17	Recover user data procedure	Recovers the user's data and request

**Table 6:** Identified trust point (TP).

TP ID	Trust point (TP)	Explanation
TP1	Remote user who is not permitted	A user who has connected to the ERP system but has not provided valid credentials yet
TP2	Remote user who is permitted	User who has certificate and has sign-in information like sign-in ID and password.
TP3	Admin	Admin uses login information to access and modify the database
TP4	Hypertext transfer protocol (HTTP) user	Hypertext transfer protocol (HTTP) is used to access the page.
TP5	Hypertext transfer protocol secure (HTTPS) user	Hypertext transfer protocol secure (HTTPS) is used to access the page.
TP6	Identification of web server process	Used to validate the web server to the database when saving or recovering information
TP7	Identification of database server process	Procedure indication is given to the accounts that used to process the DB server.

**Table 7:** Identified speculation point (SP).

SP ID	Speculation point (SP)	Explanation
SP1	e-Payment	If any responsibility is given to the e-payment, then it should not allow the hacker to hack the security features.
SP2	Payment gateway	The ERP system must co-work with any security standards that may be installed in the future
SP3	Encoded message	If any data or information is included in the ERP system, it should work properly with the encoded standards.

**Table 8:** Identified reliable point (RP).

RP ID	Reliable point (RP)	Explanation
RP1	DB server	ERP system relies on the safety of the DB
RP2	Web server	ERP system relies on the safety of the web server
RP3	Internet	ERP system relies on the safety between the web server and DB server.
RP4	External simple mail transfer protocol server	ERP system relies on the external simple mail transfer protocol server
RP5	Session administration	ERP system relies on the session administration

**Table 9:** Threats of the hospital ERP system.

TID	Threats	Explanation	STRIDE						Alleviated	VR
			S	T	R	I	D	E		
T1	User give hostile Structured Query Language (SQL) information	There is a possibility of using the application by the hacker by including the Structured Query Language		Yes				Yes	No	VR12
T2	Exposure of sign-in information	The information of sign-in details of permitted user is hacked by the hackers				Yes		Yes	No	VR2, VR3, VR4
T3	Hack of session ID	The information of session details of permitted user is hacked by the hackers						Yes	No	VR11
T4	Exposing the user information	In order to raise the privacy issue, the information of the user data will be exposed	Yes			Yes			No	VR5, VR6
T5	Entering the DB	DB of hospital ERP system will be attacked by the hacker		Yes	Yes	Yes		Yes	Yes	VR1-VR6
T6	Hacking sign in page of the admin	In the ERP system, the hacker hacks the admin page and then pretends to enter the system as the admin						Yes	Yes	VR4
T7	Notification of message is blocked	The permitted user will never receive any notification about his hack or about stealing any of his information.					Yes		Yes	VR15
T8	Falsification of user information	The information of the permitted user will be modified by the hacker	Yes	Yes				Yes	No	VR5, VR6
T9	Removing the account of the user	The account of the permitted user will be deleted by the hacker					Yes	Yes	Yes	VR2, VR3
T10	ERP system crashing	ERP web application will be crashed by the hacker					Yes		Yes	VR8
T11	Unpermitted access	Hacker hacks the sign-in information of the ERP system						Yes	Yes	VR5, VR6
T12	Entering without sign in	Information of the permitted person will be hacked without signing in			Yes				No	VR16

**Table 10:** Threats are prioritized based on their DREAD risk value.

Threat ID	Threat	DREAD value	Alleviated
T1	User give hostile structure query language (SQL) information	10	No
T5	Entering the DB	10	Yes
T10	ERP system crashing	10	Yes
T4	Exposing the user information	9.2	No
T8	Falsification of user information	9.2	No
T6	Hacking sign in page of the admin	7.6	Yes
T9	Removing the account of the user	7.6	Yes
T12	Entering without sign in	7.6	No
T2	Exposure of sign-in information	6.6	No
T7	Notification of message is blocked	6.4	Yes
T11	Unpermitted access	5.2	Yes
T3	Hack of session ID	3.8	No

**Table 11:** Security requirement of all the individual threat.

T ID	SR ID	Security requirement
T1	SR1	Use of developed statements with parameterized queries
T5	SR2	Use of entry control, checking, certification, ciphering, integrity control, backup technique
T10	SR3	Recognize the errors and update its version
T4	SR4	Encoding method is used to limit the exposure of the user information
T8	SR5	Appropriate technique and firewall is used to grant right to the permitted user
T6	SR6	Motivate user to keep creating strong passwords
T9	SR7	Strong passwords should be used for the account which has many failure attempts
T12	SR8	Virtual private network, secure sockets layer, and firewalls are used
T2	SR9	Direct Internet access by a firewall is used to protect the ERP system
T7	SR10	Guarantee the security of simple mail transfer protocol server
T11	SR11	Hard password and one-time passcode
T3	SR12	Secure sockets layer/hypertext transfer protocol secure is used to encode the ERP system

*Note*: ^*∗*^*T* means threat; SR means security requirement.

**Table 12:** Examining Model Oriented Security Requirements Engineering and Identification of Security Threats during Requirement Engineering technique.

System asset-based security requirements evoked by Model Oriented Security Requirements Engineering	
SR1	During the checking process, we should use protected checking so that it does not send the password over the Internet.
SR2	Utilize the protected communication channel.
SR3	Utilize the encoding method based on isolated process call.
SR4	Install the security system that blocks everything other than the communication ports.

System asset-based security requirements evoked by Identification of Security Threats during Requirement Engineering	

SR1	Use of entry control, checking, certification, ciphering, integrity control, and backup technique
SR2	Motivate user to keep creating strong passwords
SR3	Encoding method is used to limit the exposure of the user information
SR4	Appropriate technique and firewall is used to grant right to the permitted user

**Table 13:** Examining results of System Quality Requirements Engineering and Identification of Security Threats during Requirement Engineering technique.

Essential security requirements evoked by System Quality Requirements Engineering technology	
SQ1	Entry point should have more security
SQ2	The framework must have sufficient procedure-driven and intelligent plans to manage which framework components (information, usefulness, and so on) clients can see, adjust, and connect with.
SQ6	It is necessary that the framework's system correspondences be secured from unapproved data gathering as well as listening stealthily by encryption and other sensible methods.
SQ7	Need of prior approval for any installation to be done in the system.
SQ8	It is important to protect the asset management system (even damage due to destruction, terrorism, or acts of God/nature).

Essential security requirements evoked by Identification of Security Threats during Requirement Engineering technique (ISTDRE)	

SR1	Use of entry control, checking, certification, ciphering, integrity control, and backup technique
SR2	Motivate user to keep creating strong passwords
SR3	Encoding method is used to limit the exposure of the user information
SR4	Appropriate technique and firewall is used to grant right to the permitted user
SR5	In order to check the external security, use the HIPAA security standards.

## Data Availability

No data were used to support this study.
